The article "Alteration in Asymmetry of White Matter Network of Parkinson's Disease" was published in 2022. Journal: Contrast Media Mol Imaging.

# Alteration in Asymmetry of White Matter Network of Parkinson's Disease

**DOI:** 10.1155/2022/8493729

**Published:** 2022-07-04

**Authors:** Aihong Chen, Yue Deng, Xiaobing Zuo, Suting Zhong

**Affiliations:** ^1^Department of Emergency Medicine, Hanyang Hospital Affiliated to Wuhan University of Science, Wuhan, Hubei 430051, China; ^2^Union Hospital, Tongji Medical College, Huazhong University of Science and Technology, Wuhan, Hubei 430051, China

## Abstract

Parkinson's disease (PD) is manifest clinically by an asymmetrical presentation of motor dysfunction. A large number of previous neuroimaging research studies have stated the alteration in the hemispheric asymmetry of morphological features in PD disease. Diffusion Magnetic Resonance Imaging (MRI), which is noninvasive, has been widely used to quantify the white matter network in the human brain of both healthy subjects and patients. Besides, graph theory analysis is widely used to quantify the topological architecture of the human brain network. Lately, researchers have discovered that the topological architecture of the white matter network significantly differs in PD compared with healthy controls (HC). Nevertheless, the asymmetry of the topological architecture of the white matter network for PD patients remains unclear. To clarify this, the diffusion-weighted images and tractography technique were used to reconstruct the hemispherical white matter networks for 22 bilateral PD patients and 18 HC subjects. Network-based statistical analysis and graph theory analysis approaches were employed to estimate the asymmetry at both the connectivity level and the hemispheric topological level for PD patients. We found that the PD group showed atypically right-higher-than-left asymmetry in hemispheric brain global and local efficiencies. The detected right-higher-than-left asymmetry was driven by the atypically topological changes in the left hemispheric brain in the PD group. Findings from these studies might provide new insights into the asymmetric features of hemispheric disconnectivity and emphasize that the topological asymmetry of the hemispheric brain could be used as a biomarker to identify PD individuals.

## 1. Introduction

Parkinson's disease (PD) is a common irreversible neurodegenerative disorder in middle-aged and elderly people, involving unilateral motor symptoms in more than 85% of patients [1]. Previous neuroimaging studies reveal abnormal hemispheric asymmetry/lateralization at both structural and functional levels in PD, including lateral ventricular enlargement [2] and cortical thickness [3–6]. For example, Lewis's studies reported that there is asymmetrical lateral ventricular enlargement associated with motor asymmetry in Parkinson's disease (PD) [2]. Besides the local asymmetry for the PD, some studies reported that the abnormal hemispheric asymmetry for PD also exists at the connectivity level, such as white matter (WM) properties and functional connectivity [7–9]. Interestingly, some previous studies displayed that the left hemisphere was more sensitive than the right, suggesting that the left hemisphere might degenerate more rapidly in PD [5].

With the development of the MRI technology, the MRI-based brain “connectome” was proposed recently to model and quantify the human brain by using the complex network. Graph theory analysis approaches offer dominant ways to discover the topological architecture of the human brain connectome for both healthy and disease populations [10, 11]. Diffusion-weighted MRI, characterized by noninvasive, has been widely used to explore the white matter alteration in PD [12–15]. It is important to point out that some studies indicated altered topological properties of the WM connectome constructed by using diffusion MRI in PD. By using neuroimaging and graph theory analysis, more and more researchers agree with the notion that neurological and psychiatric disorders are caused not by abnormalities in the specific brain regions but by abnormalities in corresponding subnetworks.

So far, little is known about whether the PD patients were abnormal in the asymmetry/lateralization of hemispheric WM network topology. The main aim of this study is to explore whether there is an abnormal asymmetry of hemispheric WM network topology for the PD. Given the previously observed asymmetries in the motor dysfunction of PD patients, we proposed the hypothesis that PD patients show abnormal hemispheric network asymmetry in topological architecture. To prove this hypothesis, we used diffusion-weighted magnetic resonance imaging (dMRI) to construct the hemispheric WM network for PD patients and HC subjects. Graph theoretical analysis method, which is commonly used to quantify the topological architecture, was applied to each hemispheric brain WM network. Here, we only focus on the network efficiency-related parameters, which are usually used to quantify the network efficiency of information processing and communication.

## 2. Materials and Methods

### 2.1. Subjects

The subjects used here were reviewed by the Hanyang Hospital, Wuhan University of Science and Technology. Written informed consent has been provided by the patients/participants. The demographic information for involving subjects here is shown in Table 1. That is, a total of 22 participants with bilateral PD and 18 HC were included. There was no significant difference in either sex (*p* = 0.25) or age (*t* = 1.22; *p* = 0.23) between PD and NC participants.

### 2.2. MRI Scanning Parameters and Preprocessing Steps

The MRI data, including 3D T1 MRI and diffusion MRI, were acquired on a Philips 3T MR scanner. For each subject, 3D T1 MRI was acquired using the 3D MPRAGE sequence. The imaging parameters were 176 sagittal slices, inversion time [TI] = 1100 ms, echo time [TE] = 3.49 ms, repetition time [TR] = 7.80 ms, matrix size = 256 × 256, flip angle = 7°, and resolution = 1 × 1 × 1 mm^3^. The *T*1-weighted imaging was used for registration. The diffusion-weighted MRI was acquired using a single-short spin echo EPI sequence with the imaging parameters as followed: matrix size = 126 × 126, repetition time = 10 s, echo time = 83.47 ms, flip angle = 90°, slice thickness = 2 mm, resolution = 2 × 2 × 2 mm^3^, 32*b* = 1000 mm/s^2^ with one *b* = 0.

#### 2.2.1. Preprocessing and White Matter Network Construction for Left and Right Hemisphere

Diffusion-weighted images were preprocessed as follows. We first extracted the brain tissue and gained the brain mask. Then we corrected the distortion caused by eddy-current and the head motion of participants. The *b*-vector matrix was further readjusted by using the deformation information gained from the previous step. Finally, a diffusion tensor model was used to calculate the fractional anisotropy (FA) metrics, which is a common parameter to quantify the integration of the white matter tract. To quantify the hemispheric asymmetry, we reconstructed two hemispheric networks for each subject (Figure 1). That is the network for the left hemisphere and the right hemisphere.

To define the node of the brain network, the gray Atlas was used to separate the whole-brain gray matter into regions. Here, the previous proposed Atlas of intrinsic connectivity of homotopic areas (AICHA) [16] was used, considering that the AICHA Atlas thinks about the regional homotopy between two hemispheres when separating the gray matter regions. According to the Atlas, the hemispheric brain gray matter was divided parcellated into 192 cerebral regions (including 170 cortical regions and 22 subcortical gray matter regions).

For each subject, we performed whole-brain fibre tractography using the fibre assignment by continuous tracking algorithm (FACT for short) [17], which is one of the most commonly used deterministic tractographies, using the TrackVis Diffusion Toolkit (trackvis.org). The fibre tracking terminated when it entered the voxels whose FA value was less than 0.2 or the angle between adjacent two steps was higher than 45°. In this study, the mean FA values were used as the edge weight. As an important index to quantify fibre integrity [18], FA has been widely used as a candidate to quantify the efficiency of brain connections [19, 20]. For each subject, two hemispheric 192 × 192 symmetric FA-weighted matrices were finally constructed.

As the gray Atlas mentioned above is in the MNI standard space, and the tractography is in the individual space. In order to match the node and the edge of the network, we transformed the gray Atlas into the individual space by the following steps. First, we realigned the T1-weighted images to the FA images, resulting in a transform matrix. Then, we realigned the individual *T*1-weighted images to the *T*1-weighted images in the MNI standard space, resulting in a transformed image. Finally, the results of the previous two steps were used on the gray Atlas, and we got the individual parcellation.

### 2.3. Network Topological Metrics

To quantify the topological properties of hemispheric brain white matter networks, the graph theory was used to calculate the efficiency-related metrics [10]. More specifically, we calculated the network global efficiency (Eg) and network local efficiency (El) to characterize the information communication efficiency at the whole hemispheric brain level. Besides, the nodal efficiency (En) was computed for each node/region [21]. We described these network metrics briefly as follows:

#### 2.3.1. Global Efficiency Metrics at Hemispheric Level

Hemispheric global network efficiency (Eg) is a hemispheric brain metric defined as the mean inverse shortest path length [22] of a hemispheric network. Eg quantified the average ability of information communication at the whole hemispheric brain level. The larger the Eg is, the more powerful the efficiency is.

#### 2.3.2. Local Efficiency Metrics at Hemispheric Level

Hemispheric local efficiency (El) is also a hemispheric brain level metric which is defined as the mean/average of the nodal local efficiencies of a hemispheric brain network [22]. El quantified the average efficiency of information communication within the focal regions and is usually used to reflect the average capacity of a network to accept faults.

### 2.4. Nodal Efficiency Metrics at Hemispheric Level

Hemispherical node efficiency of a certain node *i* (En) is definite as the average of the shortest path length of the node *i* and all left nodes (191 nodes, a total of 192 nodes for each hemisphere) in the hemispheric network [23]. En indicates the ability of a node to communicate with other nodes in the hemispheric brain network.

All the topological metrics were computed by using GRETNA2 [21].

### 2.5. Hemispheric Asymmetry Index (AI)

We used the commonly used asymmetry index (AI), which was computed by using the following formula, to evaluate the degree of hemispheric differences:

(1) $$\begin{array}{c} \text{AI}=\frac{\left(R-L\right)}{\left(\left(R+L\right)/2\right)}. \end{array}$$

Here, for the network topological architecture, *R* and *L* stand for the abovementioned hemispheric efficiency-related metrics of right and left hemispheric networks. At the connectivity level, the *R* and *L* stand for the connectivity weights (FA value) for each connectivity. According to the formula, positive and negative AI denote a leftward and rightward asymmetry, respectively.

#### 2.5.1. Statistical Analysis Methods

In this study, we used a proven method named network-based statistics (NBS) proposed by Zalesky et al. [24] to recognize the subnetworks (known as network components with brain regions and connections between these regions) whose edges were significant differences between two dslqgroups on the asymmetry index of the connectivity weights. More specifically, the nonparametric permutation test was used and the input for the NBS analysis was the FA-weighted undirected connectivity matrices gotten from deterministic tractography. The connectivity significant level was set to 0.01 and the null distribution was generated by 10000 permutations. The networks showing group effects on the asymmetry index of the connectivity between regions (FA value) with a significance of *p* < 0.05 were reported.

At the topological level, we first tested the asymmetries of topological parameters (i.e., hemispheric network global efficiency [Eg], hemispheric network local efficiency [El], and hemispheric nodal efficiency [En]) for each group (i.e., PD and HC). Here, repeated general linear models were used. In detail, the left and right hemispheric regions of the brain were considered as the repeated variables; age and sex were used as covariates. Besides, we explored the group differences in topological efficiency using a general linear model with AI of topological efficiency as the dependent variable and the group as the independent variable. For whole-level network efficiencies (i.e., Eg and El), the significant level was set to 0.05. For the nodal level efficiency metrics, FDR multiple-comparison correction was performed, and the corrected significant level was set to *q* < 0.05.

## 3. Results

### 3.1. Subnetwork with Altered White Matter Connectivity Asymmetry

We employed the NBS to recognize a subnetwork (network components). These network components contained 76 nodes/regions and 88 connections. Those connections were significantly white matter connectivity asymmetry altered in the patients (*p* = 0.025, as shown in Figure 2(a)). The nodes are listed in Table 2. This subnetwork mainly included the middle temporal gyrus (6 connections), the inferior part of the temporal gyrus (6 connections), the superior frontal gyrus (5 connections), the supramarginal gyrus (5 connections), the angular gyrus (5 connections), and the middle occipital gyrus (5 connections) (as shown in Table 2). Further analysis indicated that the subnetwork is significant leftward for the HC group (*t* = −18.44, *p* < 0.0001) but significant rightward for the PD group (*t* = 24.99, *p* < 0.0001, Figure 2(b)).

### 3.2. The Hemispheric Effects on the Network Efficiencies for Each Group

The hemispheric effects on the hemispheric network efficiencies for both PD patients and the HC group are illustrated in Figure 3. Both the Eg and El were explored. We found that both the PD group and the HC group were significantly rightward asymmetry in global network efficiency (For HC group: *F* = 2.26, *P* = 0.045; For PD group: *F* = 3.09, *P* = 0.0067). For network local efficiency, we found that there were no significant hemispheric effects in the HC group (*F* = 0.1522, *P* = 0.88), but significant rightward asymmetry for the PD group (*F* = 2.38, *P* = 0.027).

### 3.3. Group Effects on the Hemispheric Differences

In this study, the sex-group interaction effect on either the asymmetry index of El (*F* = 1.95; *P* = 0.195) or the asymmetry index of Eg (*F* = 2.27; *P* = 0.14) was not significant, indicating the similar group difference in both female and male subjects.

We explored the group difference after removing the sex-group interaction term from the general linear model, considering no sex-group interaction. The group differences on the AI of Eg (*F* = 4.34; *P* = 0.045) were found to be significant. We further checked the group effects for each hemispheric brain and we found that two groups (PD and HC) had significant differences in left hemispheric global efficiency but not in that of the right hemisphere (Eg LH: *F* = 4.32, *P* = 0.045; Eg RH: *F* = 0.08; *P* = 0.76; Figure 4(a), LH means left hemisphere, RH means right hemisphere).

For hemispheric El, there were significant differences in the asymmetry index (*F* = 5.177; *P* = 0.0291) between the PD and HC groups. For the left hemispheric brain, there were significant group differences in network local efficiency (El) (El of left hemisphere: *F* = 4.30, *P* = 0.047). For network local efficiency of the right hemisphere, there was no significant group difference (El of the right hemisphere: *F* = 0.58; *P* = 0.45; Figure 4(b)). Compared with the HC group, the increase in right asymmetry in the PD group may be mainly due to the reduction of overall network efficiency in the left hemisphere in the PD group.

### 3.4. Hemispheric Effect on the Nodal Efficiency for Each Group

Figure 4 exhibits the nodes/regions with significant hemispheric effects on the En (FDR-corrected *P* < 0.05) for each group. There were 12 significant leftward nodes (192 in all) and 79 significant rightward nodes in the NC group. For the PD group, we found 14 significant rightward asymmetry nodes and 59 nodes with significant leftward asymmetry in nodal efficiency. For the HC group, the regions/nodes showing left-higher-than-right nodal efficiency were mostly located in the supramarginal gyrus and intraparietal sulci, while the regions/nodes showing right-higher-than-left nodal efficiency were found in the temporal pole, amygdala, postcentral gyrus, middle part of the temporal pole, thalamus, supplementary motor area, cingulum, caudate, supramarginal gyrus, superior temporal gyrus, superior medial frontal gyrus, and superior frontal gyrus (as shown in Figure 5 and Table 3). For the PD group, the regions/nodes showing left-higher-than-right nodal efficiency were mostly located in the middle frontal gyrus and posterior insular gyrus, while the regions/nodes showing right-higher-than-left nodal efficiency were found in the superior temporal gyrus, caudate, parahippocampal, and hippocampus (as shown in Figure 5(b) and Table 4).

### 3.5. Abnormal Asymmetry of Nodal Efficiency in PD Group

As shown in Figure 6, a significant difference between PD and HC subjects in the asymmetry index of hemispheric En was found. The nodal efficiency of 11 nodes (*P* < 0.05 uncorrected; 192 in total) was a significant group difference in the degree of asymmetry. The nodes with significant group effects on AI were mainly the parahippocampal gyrus, inferior temporal gyrus, orbitofrontal cortex, precuneus, superior parietal gyrus, thalamus, cingulate, and temporal pole (Table 5, Figure 6).

## 4. Discussion

In this study, we explored alterations in the asymmetry for PD patients between the left and right hemispheres at the network level. The core discoveries are follows: (1) the white matter network in the hemispheric brain of PD patients exhibits an abnormal right-higher-than-left topological asymmetry; (2) only the topological properties of the left hemisphere show significant between-group differences, suggesting that the left hemisphere has an abnormal topology in PD; and (3) compared with normal controls, the degree of asymmetry of lymph node efficiency in PD patients to the right is mainly around the temporal lobe. Our findings provide direct evidence for the change of network asymmetry in patients with Parkinson's disease and expand our understanding of the neurophysiological mechanism of Parkinson's disease from the perspective of network asymmetry.

Previous whole-brain network studies showed that PD patients presented reduced efficiency [25, 26]. Our study found comparable results at the cerebral hemisphere level. Specifically, we found that the network efficiency was significantly reduced in the left hemisphere of PD patients compared with HC subjects. Our findings are consistent with previous findings [5]. In all, these results support the long-term view that PD is a disconnection syndrome [27].

Additionally, we found that HC subjects showed left-higher-than-right network efficiency, which indicates that the information exchange efficiency in the left hemisphere is significantly higher than in the right hemisphere for HC subjects. This finding is inconsistent with previous studies. For example, Yang et al. [28] reported that the HC subjects showed a symmetric network efficiency. This inconsistency may be caused by the difference in network size. As shown in previous studies, the network size is an influencing factor in topology metrics of white matter networks [29]. Yang et al. (2017) [28] involved 512 nodes (high resolution), while 192 nodes (relatively low resolution) were used in this study.

What is noteworthy is that the hemispheric network efficiency of PD patients showed significant rightward asymmetry, which indicates that the regions in the left hemisphere are connected by white matter in a worse integrated way, and the communication efficiency of the left hemisphere is lower at the hemispheric level of PD. These results are generally consistent with early studies, that is, the left hemisphere of PD patients loses GM faster than the right hemisphere [5].

## 5. Conclusion

Based on diffusion-weighted imaging and tractography, we found that the PD patients showed increased rightward asymmetry in hemispheric brain white matter networks, and the rightward asymmetry is derived from the abnormalities of the left hemisphere. In addition, the alteration asymmetry can be found both at the connectivity level and at the topological level. These findings provide insights into the pathological mechanisms of PD and unlock the potential of brain network-based biomarkers for PD.

## Figures and Tables

**Figure 1:** Diagram of intrahemispheric WM connections. Whole-brain fibres were estimated using a deterministic tractography technique. The AICHA Atlas was applied to separate the hemispheric cerebral gray matter into 192 regions [16].

**Figure 2:** The white matter connections, which display significant asymmetries in connectivity weights.

**Figure 3:** The difference in the hemispheric network global and hemispheric network local efficiency between the right and left hemispheres for both the HC group and the PD group. (a) Hemispheric network Eg; (b) Hemispheric network El. Notably, the general linear model was conducted with age, sex, and education as confounding factors. ^∗^ specifies significant hemispheric effects (*P* < 0.05).

**Figure 4:** Group differences in the network global efficiency （Eg） and network local efficiency（El） in the two hemispheres. (a) Eg; (b) El. Notably, the general linear model was conducted with age, sex, and education as confounding factors. ^*∗*^ means a significant asymmetry (*P* < 0.05).

**Figure 5:** The asymmetry index map of the nodal efficiency for both the HC group and the PD group. (a) The AI map for the PD group; (b) the significant hemispheric effects on the nodal efficiency for the PD group; (c) the AI map for the HC group; (d) the significant hemispheric effects on the nodal efficiency for the HC group.

**Figure 6:** The group difference in asymmetry index between the HC and PD groups. The general linear model was conducted with age, sex, and education as confounding factors.

**Table 1:** Demographic information of study participants.

	Number of subject	Age (Mean ± std)	Sex (F/M)
HC	18	65.63 ± 10.33	8/10
PD	22	62.71 ± 10.39	6/16
*P* value	-	0.23	0.25

**Table 2:** Regions which showed significant group effects on the asymmetry of the white matter connectivity weight.

Regions	Number of edges
Gyrus_Temporal_Middle-4	6
Gyrus_Temporal_Inferior-5	6
Sulus_Superior_Frontal-4	5
Gyrus_Supramarginal-3	5
Gyrus_Angular-3	5
Gyrus_Occipital_Middle-3	5
Sulus_Superior_Frontal-5	4
Gyrus_Frontal_Middle-4	4
Sulus_Postcentral-2	4
Sulus_Superior_Temporal-3	4
Sulus_Superior_Frontal-3	3
Gyrus_Parietal_Superior-1	3
Gyrus_Parietal_Superior-4	3
Gyrus_Supramarginal-4	3

**Table 3:** Regions/nodes with significant hemispheric difference on nodal efficiency for the HC group.

	Region name	*F* value
HC leftward	Gyrus_SupraMarginal-5	4.648
	Sulus_Intraparietal-1	4.130

HC rightward	Gyrus_Cingulum_Post-1	5.759
	Nuclei_Thalamus-4	5.943
	Nuclei_Caudate-5	6.209
	Sulus_Superior_Frontal-4	6.534
	Gyrus_Frontal_Superior_Medial-1	6.589
	Gyrus_Temporal_Superior-3	7.197
	Gyrus_SupraMarginal-7	7.296
	Nuclei_Caudate-4	7.466
	Gyrus_Cingulum_Mid-1	7.504
	Gyrus_Superior_Motor_Area-3	8.494
	Nuclei_Thalamus-3	8.540
	Gyrus_Temporal_Pole_Middle-1	8.822
	Nuclei_Thalamus-9	9.489
	Sulus_Postcentral-3	9.516
	Nuclei_Amygdala-1	9.910
	Gyrus_Temporal_Pole_Superior-1	14.723

**Table 4:** Regions/nodes with significant hemispheric difference on the nodal efficiency for PD group.

	Region name	*F* value
PD leftward	Gyrus_Frontal_Middle-5	7.129
	Gyrus_Insula-Posterior-1	5.149
	Gyrus_Frontal_Middle-3	5.049

PD rightward	Gyrus_Temporal_Superior-3	6.402
	Nuclei_Caudate-4	6.691
	Gyrus_ParaHippocampal-1	6.873
	Gyrus_Hippocampus-1	7.129
	Nuclei_Thalamus-9	7.773
	Gyrus_Superior_Motor_Area-3	8.131
	Gyrus_Temporal_Middle-1	9.321
	Gyrus_Temporal_Pole_Superior-1	9.508
	Sulus_Postcentral-3	11.146
	Gyrus_Temporal_Pole_Middle-1	11.693
	Nuclei_Amygdala-1	13.132

**Table 5:** Regions/nodes with significant group differences in the asymmetry index (AI) of En (nodal efficiency).

	Region name	*F* value
Group differences in AI	Gyrus_ParaHippocampal-1-L	11.065
	Gyrus_Temporal_Inf-3-L	9.651
	Gyrus_Frontal_Superior_Orb-1-L	8.750
	Gyrus_Precuneus-7-L	8.579
	Gyrus_Parietal_Superior-3-L	6.193
	Gyrus_Frontal_Med_Orb-2-L	5.939
	Nuclei_Thalamus-1-L	4.896
	Sulus_Cingulate-2-L	4.821
	Gyrus_Temporal_Pole_Mid-2-L	4.552
	Gyrus_Precuneus-1-L	4.405
	Gyrus_Parietal_Sup-1-L	4.278

## Data Availability

The data used to support the findings of this study are available from the corresponding author upon request.
